This article has been retracted.

# Downregulating lncRNA NEAT1 induces proliferation and represses apoptosis of ovarian granulosa cells in polycystic ovary syndrome via microRNA-381/IGF1 axis

**DOI:** 10.1186/s12929-021-00749-z

**Published:** 2021-07-15

**Authors:** Jingran Zhen, Jiangli Li, Xia Li, Xue Wang, Yaling Xiao, Zhengyi Sun, Qi Yu

**Affiliations:** 1 Department of Gynecological Endocrinology and Reproduction Center, Peking Union Medical College Hospital, Chinese Academy of Medical Sciences, 41 Damucang Hutong, Xicheng, Beijing, China; 2 Department of Obstetrics and Gynecology, Zhongguancun Hospital, Beijing, 100080 China; 3 Community Health Service Center, Beijing Forestry University, Beijing, 100053 China

**Keywords:** Polycystic ovary syndrome, Long non-coding RNA nuclear-enriched abundant transcript 1, MicroRNA-381, Insulin-like growth factor 1, Ovarian granulosa cells, Apoptosis, Proliferation

## Abstract

**Objective:**

Researchers have revealed the combined functions of long noncoding RNAs (lncRNAs) and microRNA (miRNAs) in polycystic ovary syndrome (PCOS). This study aimed to understand the role of nuclear-enriched abundant transcript 1 (NEAT1) and miR-381 involving insulin-like growth factor 1 (IGF1) in PCOS.

**Methods:**

PCOS rat model was established by dehydroepiandrosterone induction. NEAT1, miR-381 and IGF1 expression in ovarian granulosa cells of PCOS patients and ovarian tissues of PCOS rats were tested. Bioinformatics website and dual luciferase reporter gene assay were utilized to verify the relationship between NEAT1 and miR-381 and that between miR-381 and IGF1. Levels of sex hormone, pathological changes and ovarian granulosa cell apoptosis in ovarian tissues of PCOS rats were detected. Ovarian granulosa cell proliferation and apoptosis were analyzed in vitro.

**Results:**

NEAT1 and IGF1 expression increased while miR-381 expression decreased in the ovarian granulosa cells of patients with PCOS and the ovarian tissues of PCOS rats. In in vivo experiments, interference with NEAT1 improved the levels of sex hormones, alleviated pathological changes and suppressed ovarian granulosa cell apoptosis in the ovarian tissues of PCOS rats. In in vitro cell experiments, interference with NEAT1 suppressed apoptosis and enhanced cell proliferation of ovarian granulosa cells. NEAT1 interference-mediated effect would be reversed by up-regulating miR-381. NEAT1 acted as a ceRNA to adsorb miR-381 to target IGF1. Overexpression of IGF1 reversed the inhibitory effect of miR-381 on ovarian granulosa cell apoptosis.

**Conclusion:**

Interference with NEAT1 increases miR-381 and reduces IGF1 levels, effectively improving the levels of sex hormones and reducing the pathological damage of ovarian tissue in rats with PCOS.

**Supplementary Information:**

The online version contains supplementary material available at 10.1186/s12929-021-00749-z.

## Introduction

Polycystic ovary syndrome (PCOS) is a reproductive endocrine disease that is often characterized by increased dehydroepiandrosterone (DHEA) [1, 2]. PCOS affects 5–10% of women at reproductive age and generally is featured by oligo/anovulatory cycles, hirsutism and polycystic ovaries, together with a considerable prevalence of insulin resistance [3]. Up-regulated luteinizing hormone levels are thought to contribute to high androgen levels, and increased androgen levels have an adverse effect on follicular development. Retardation of endogenous luteinizing hormone secretion by antagonists and ovulation induction could facilitate follicular development theoretically [4]. At present, exploring effective agents is urgently required for the treatment of PCOS.

Long non-coding RNAs (lncRNAs) are non-coding RNA transcripts that participate in the pathogenesis of PCOS [5, 6]. Of the lncRNA family, nuclear-enriched abundant transcript 1 (NEAT1) has been revealed to regulate ovarian carcinogenesis and act as a potential biomarker for antineoplastic therapies [7, 8]. Moreover, NEAT1 has the ability to promote ovarian granulosa cell proliferation and suppress apoptosis through acting as a sponge of microRNAs (miRNAs) [9]. miRNAs that are differentially expressed in PCOS are related to the pathophysiology of the disease [10]. For example, repressed miR-129 expression could induce endocrine disturbance, suppress proliferation and enhance apoptosis of ovarian granulosa cells in PCOS [11]. According to miRNA ChIP analysis, it is shown that miR-381-3p is related to the progression of PCOS [12]. However, the specific mechanism of miR-381 has not been explored. Therefore, miR-381 was selected for research out of innovation. Insulin-like growth factor 1 (IGF1) was predicted as a target gene of miR-381 on the online website of our research. Specially, IGF1 is one of the highly expressed genes in PCOS that contribute to the aggravated endocrine disorder and granulosa cell apoptosis [13]. There is a recent study confirming that overexpressed IGF1 is associated with early miscarriage in PCOS patients [14]. Another study has revealed that the concentration of IGF1 is high in follicular fluid of patients with PCOS [15]. However, the potential mechanism of NEAT1/miR-381/IGF1 axis in PCOS has not been explored yet. Therefore, this research was determined to grasp the mechanism of NEAT1 in ovarian granulosa cell proliferation and apoptosis with the involvement of miR-381 and IGF1 in PCOS.

## Materials and methods

### Ethics statement

The study was agreed by the Ethics Committee of Peking Union Medical College Hospital (ethics number: 201601203). The participants signed the written informed consent. The study was agreed by the Animal Ethics Committee of Peking Union Medical College Hospital (ethics number: 201601214). All animal experiments were conducted in line with the Guide for the Care and Use of Laboratory Animal of National Institutes of Health.

### Clinical data

Patients with PCOS (n = 92) in Peking Union Medical College Hospital were enrolled in the PCOS group (average age of 28.21 ± 5.26 years). At the same time, infertile patients (n = 108) with fallopian tube-related diseases were enrolled in the non-PCOS group (average age of 27.26 ± 4.88 years). PCOS was diagnosed according to the PCOS diagnostic standard in 2003 [16]. Patient were excluded if they had hyperandrogenism caused by other diseases (such as congenital adrenal hyperplasia, Cushing syndrome) or had administrated with hormone drugs in the past 3 months. The non-PCOS patients had regular menstrual cycles, dual-directional thermoregulation without ovarian physiological cysts, corpus luteal cysts, ovarian tumors or administration of hormone drugs in the past 3 months. All patients were treated with GnRH agonists and recombinant follicle stimulating hormone (150 187.5 IU; Gonal-f, Follitropin Alfa, Serono). When two or more follicles were grown to at least 18 mm, 250 μg of human chorionic gonadotropin (HCG) (Profasi; Serono) was administrated. At 36 h post HCG administration, the follicular fluid from the follicle (18 mm) was extracted by vaginal ultrasound, centrifuged, mixed with 50% percoll solution (Transtech, Beijing, China) and treated with centrifugation to collect the granulosa cells. Cells were cultured in Dulbecco’s modified Eagle medium (DMEM) with 10% fetal bovine serum (FBS), 100 IU/mL penicillin and 100 μg/mL streptomycin (BD Biosciences, San Jose, CA). The prospective cohort study was conducted in Peking Union Medical College Hospital from April 2017 to April 2019. The clinical data were shown in Table 1.

**Table 1:** Clinicopathological features

Parameters	Non-PCOS (n = 108)	PCOS (n = 92)	*P*
Age	27.26 ± 4.88	28.21 ± 5.26	0.187
BMI	23.12 ± 3.60	24.19 ± 5.03	0.082
Basal antral follicle count	14.27 ± 3.58	27.28 ± 6.21	< 0.001
Basal E2 (pg/ml)	42.45 ± 17.38	56.14 ± 20.86	< 0.001
Basal testosterone (nmol/ml)	0.98 ± 0.52	1.78 ± 0.86	< 0.001
Basal FSH (mlU/ml)	6.91 ± 2.92	5.70 ± 2.27	0.002
Basal LH (mlU/ml)	4.63 ± 2.47	8.39 ± 5.35	< 0.001

### Experimental animals

Wistar female rats (7–8 w, 220–260 g, Laboratory Animal Center of Peking Union Medical College Hospital, Beijing, China) were fed for a week in an environment of clean grade (no zoonotic pathogens, severe infectious disease pathogens, common infectious disease pathogens, or pathogens that may carry great harm to animals and interfere with the research). The rats were housed at 20–25 °C with 55–60% humidity, 12 h day/night cycle and enough food and drinking water.

### PCOS induction and grouping

PCOS was induced according to some previous articles [17–19]. Wistar female rats were subcutaneously injected with DHEA (6 mg/100 g, Wuhan Huamei Technology Group Co., Ltd., Wuhan, China) into the back and neck (once a day for 20 d). By examining the vaginal cytology for 10 d for estrous cycle, plasma hormonal profiles and ovarian histological examinations [20], 28 PCOS rats were successfully induced. Eight healthy Wistar rats were used in the normal group and only injected with oiling reagent at 0.2 mL/d.

Twenty-four PCOS rats were randomly divided into 3 groups (n = 8/group): the DHEA group, the short hairpin RNA (shRNA)-negative control (NC) group and the sh-NEAT1 group. Rats in the DHEA group, sh-NC group and sh-NEAT1 group were fasted for 12 h. After anesthesia, rats were fixed in a supine position and injected with normal saline, shRNA-NC or NEAT1-shRNA vector (GenePharma Co, Ltd., Shanghai, China) into the ovary [21]. At 30 d post injection, rats were fasted for 12 h and their caudal vein bloods were collected, centrifuged and stored at − 80 °C.

### Detection of sex hormones

The caudal vein blood from rats was used to detect estradiol (E2), progesterone (P4), testosterone (T), follicle stimulating hormone (FSH) and luteinizing hormone (LH) by enzyme-linked immunosorbent assay (ELISA) kit (Beckman Coulter Life Sciences, Brea, CA, USA).

### Sample collection

Thirty days after injection, the rats were euthanized by cervical dislocation. The laparotomy was performed in an aseptic condition to accurately extract the bilateral ovaries and remove excess fat connective tissues around the ovary. A part of tissues was fixed in 4% paraformaldehyde (24 h) for hematoxylin–eosin (HE) staining and terminal deoxynucleotidyl transferase-mediated 2′-deoxyuridine 5′-triphosphate nick end-labeling (TUNEL) staining. The other part of tissues was stored in liquid nitrogen for gene expression analysis.

### HE staining

The ovarian tissues were fixed in 4% paraformaldehyde for 24 h, embedded in paraffin, cut into 6-μm sections, and stained with hematoxylin and eosin for 10 min. The sections were differentiated using 1% hydrochloric acid alcohol for 10 s, rinsed with 2% sodium bicarbonate for 10 s and stained with eosin for 3 min. Then, the sections were dehydrated with gradient alcohol, cleared with xylene, and sealed with neutral resin. After that, the sections were observed and photographed. Five slices were taken from every ovary, and the number of corpus luteum and mature follicles was counted.

### TUNEL assay

TUNEL kit (Nanjing KeyGen Biotechnology Co. Ltd., Nanjing, China) was applied for cell apoptosis detection. The ovarian tissues (fixed in 4% paraformaldehyde for 24 h) were dewaxed, hydrated and treated with proteinase K. The tissues were added with TdT enzyme working solution, reacted with horseradish peroxidase working solution, developed with diaminobenzidine, counter-stained by hematoxylin and observed under a microscope. Cells with brown-yellow particles in the nuclei were the positive cells. Three fields were randomly taken under the microscope, and the apoptotic index (the number of positive cell/the number of total cells × 100%) was calculated.

### Subculture of ovarian granulosa cells

PCOS rats were euthanized by cervical dislocation 2 days after modeling, and their ovarian tissues were placed in normal saline. The ovarian surface envelope and surrounding adipose tissues were removed under a microscope, erythrocytes on the surface were washed with normal saline and the ovarian tissues were placed in serum-free DMEM/F12 (Gibco, Carlsbad, California, USA). A 1-mL syringe needle was used to pierce the follicle, and the follicular granulosa cells were released. Next, follicular granulosa cells were filtered through a 200-mesh sieve and centrifuged (1000 r/min, 8 min). Then, the pelleted granulosa cells were cultured in DMEM/F12 containing 15% FBS (37 ℃; 5% CO_2_). The medium was exchanged 24 h later and the adherent cells were removed. When the cell confluence reached 80% or more, cells were detached by 0.25% trypsin and passaged. Ovarian granulosa cells were identified by HE staining and immunochemistry of follicle stimulating hormone receptor (FSHR).

### Grouping and transfection of ovarian granulosa cells

The ovarian granulosa cells from PCOS rats were divided into 10 groups: the blank group, sh-NC group (transfected with shRNA-NC), sh-NEAT1 group (transfected with NEAT1-shRNA), mimic NC group (transfected with scrambled miRNA mimic), miR-381 mimic group (transfected with miR-381 mimic), pc-NEAT1 + mimic NC group (transfected with pcDNA-NEAT1 and scrambled miRNA mimic), pc-NEAT1 + miR-381 mimic group (transfected with pcDNA-NEAT1 and miR-381 mimic), pc-CON + mimic NC group (transfected with pcDNA-IGF1-NC and scrambled miRNA mimic), pc-IGF1 + mimic NC group (transfected with pcDNA-IGF1 and scrambled miRNA mimic) and pc-IGF1 + miR-381 mimic group (transfected with pcDNA-IGF1 and miR-381 mimic). shRNA-NC, NEAT1-shRNA, mimic NC, miR-381 mimic, pcDNA-NC, pcDNA-NEAT1, pcDNA-CON and pcDNA-IGF1 were synthesized by GenePharma.

The cells were seeded in a 12-well plate 24 h before transfection, and cultured with 1.5 mL of complete penicillin/streptomycin-free medium to reach 80% confluence. Ovarian granulosa cells were transfected via Lipofectamine 2000 (Invitrogen, Carlsbad, CA, USA), and the culture solution was replaced after 6 h. The cells after 48-h culture were collected for subsequent experiments.

### Reverse transcription quantitative polymerase chain reaction (RT-qPCR)

Total RNA in tissues and cells was extracted by the RNA extraction kit (Invitrogen). The primers were designed by Takara Biotechnology Ltd. (Dalian, China) with U6 and glyceraldehyde phosphate dehydrogenase (GAPDH) as the internal controls (Table 2). The RNA was reversely transcribed into cDNA by PrimeScript RT kits. RT-qPCR was conducted in the ABI PRISM® 7300 system with SYBR® Premix Ex Taq™ II kits. Target gene levels were calculated by 2^−ΔΔCt^ method.

**Table 2:** Primer sequence

Gene	Primer sequence
miR-381	F: 5′ TGGTACTTAAAGCGAGGTTGC 3′
	R: 5′ GGTCATGCACACACATACCAC 3′
U6	F: 5′ CTCGCTTCGGCAGCACATATACT 3′
	R: 5′ ACGCTTCACGAATTTGCGTGTC 3′
NEAT1	F: 5′ TGGCTAGCTCAGGGCTTCAG 3′
	R: 5′ TCTCCTTGCCAAGCTTCCTTC 3′
IGF1	F: 5′ CTCTTTCTACCTGGCGCTCTG 3′
	R: 5′ GCAACACTCATCCACAATGC3′
PCNA	F: 5′ GATGTTCCTCTCGTTGTGGAG3′
	R: 5′ CATTGCAGTTAAGAGCCTTCC3′
Cyclin D1	F: 5′ AGCTGAGGCGTCCCAACC 3′
	R: 5′ CAACCAGAATACACAAAGCCAACC 3′
Caspase-3	F: 5′ GACTAGCTTTCTTCAGAGGCGA 3′
	R: 5′ ATTCCGTTGCCACCTTCCTG3′
Bax	F: 5′ CTGCAGAGGATGATTGCTGA 3′
	R: 5′ GATCAGCTCGGGCACTTTAG 3′
Bcl-2	F: 5′ CGACTTTGCAGAGATGTCCA3′
	R: 5′ ATGCCGGTTCAGGTACTCAG3′
GAPDH	F: 5′ ACGGCAAGTTCAACGGCACAG 3′
	R: 5′ GACGCCAGTAGACTCCACGACA 3′

*F* forward, *R* reverse, *MiR-381* microRNA-381, *IGF1* insulin-like growth factors-1, *PCNA* proliferating cell nuclear antigen, *Bax* B-cell lymphoma 2-associated X, *Bcl-2* B-cell lymphoma 2, *GAPDH* glyceraldehyde-3-phosphate dehydrogenase

### Western blot analysis

Tissue samples (15–20 mg) were placed in the centrifuge tube, ground 50–60 times with a plastic stick, added with 200 μL of natural cell lysate and ground 30–60 times. The samples were incubated on ice for 5 min and centrifuged at 14,000–16,000 rpm at 4 °C for 1–2 min. Then, the tube was placed on ice, and protein was collected. Protein concentration was determined by a bicinchoninic acid kit (AmyJet Scientific, Wuhan, Hubei, China). The extracted protein was separated by 10% polyacrylamide gel electrophoresis and transferred to a nitrocellulose membrane. The membrane was blocked by 5% skim milk and incubated with primary antibodies IGF1 (1:1000), caspase-3 (1:500), Cleaved caspase-3, Bax, Bcl-2, and GAPDH (1:1000, Cell Signaling Technology, Beverly, MA, USA). After that, the membrane and the secondary antibody (1:5000; Thermo Fisher Scientific) were incubated for 1 h and the protein bands were visualized by the enhanced chemiluminescence kits (Pierce, Rockford, IL, USA). GAPDH was the internal control and protein band images were analyzed by ImageJ2x V2.1.4.7 (Rawak Software, Inc., Germany). This method is also suitable for cell experiments.

### Cell counting kit-8 (CCK-8) assay

After transfection, the cells were cultured for 48 h and detached with 0.25% trypsin. Cells were seeded in a 96-well plate at 3000 cells (100 μL/well) and incubated. Next, 10 μL of CCK-8 reagent (Sigma-Aldrich Chemical Company, St Louis MO, USA) was added to each well at 24 h, 48 h, and 72 h, respectively, and incubated with the cells for another 4 h. The optical density (OD_490 nm_) value was read on a microplate reader (Jijia Intelligent Technology Co., Ltd., Wuxi, China).

### Colony formation assay

Cells were cultured in 12-well plates (3 × 10^3^ cells/well) and cultured for 7 days. After that, cells were fixed with 10% neutral formalin for more than 4 h, followed by staining with crystal violet solution (Beyotime, Shanghai, China) and observation under a microscope (Olympus, Tokyo, Japan).

### Flow cytometry

Ovarian granulosa cells were transfected for 48 h, trypsinized, resuspended in PBS repeatedly and fixed by pre-cooled 70% ethanol overnight. Cells were mixed with Annexin V-labeled protein (Beyotime Biotechnology Co., Shanghai, China) and the corresponding nucleic acid dye. The cells were resuspended in 1 × binding buffer (400 μL, a liquid that is used to increase the binding activity of the elution column to nucleic acids) and detected on a flow cytometer (NovoCyte Penteon, Agilent, China). The data were analyzed by Windows 3.0 software (Beckman Coulter Life Sciences).

### Dual luciferase reporter gene assay

NEAT1 wild type (WT) or that containing mutated binding sites of miR-381 (mutant, Mut) was cloned into the pmirGLO vector (Promega, WI, USA) to generate pmirGLO-NEAT1-WT/Mut plasmid. IGF1 3′-untranslated region (UTR) containing the binding site (WT) or that containing the mutated binding site (Mut) was also cloned into the pmirGLO vector to produce pmirGLO-IGF1-WT/-Mut plasmids. Cells were co-transfected with pmirGLO-NEAT1-WT/Mut or pmirGLO-IGF1-WT/Mut and miR-381 mimic or mimic NC. After transfection, the luciferase activity was measured by a Dual-Luciferase Reporter Assay System (Promega).

### RNA-pull down assay

Biotinylated miR-381 WT and miR-381 Mut were transfected into ovarian granulosa cells. After treated with the lysis buffer (20 mM Tris–HCl, 50 mM NaCl, 5 mM ethylene diamine tetraacetic acid and 0.1% Triton-X100), cells were incubated with M-280 streptavidin magnetic beads (Sigma-Aldrich) pre-coated with RNase-free and yeast tRNA (Sigma-Aldrich) and rinsed with low salt buffer (0.5 M NaCl, 0.05 mM Tris–HCl and 0.01 M MgSO_4_) and high salt buffer (1 M NaCl, 10 mM Tris–HCl and 0.1 mM ethylene diamine tetraacetic acid). The bound RNA was extracted by Ttrizol reagent (Thermo Fisher Scientific) and NEAT1 expression was detected by RT-qPCR.

### Statistical analysis

Data were analyzed by SPSS 21.0 software (IBM Corp. Armonk, NY, USA). The measurement data were expressed as mean ± standard deviation. Data were evaluated by *t*-test (two groups) or one-way analysis of variance (ANOVA) followed by Tukey’s post hoc test (multiple groups). Pearson analysis was used for correlation analysis. Statistical significance was set at *p* < 0.05.

## Results

### High expression of NEAT1 and IGF1, and low expression of miR-381 are found in patients with PCOS

NEAT1 is involved in the progression of human diseases by regulating miRNAs [22], but its function in PCOS is unclear. In this study, NEAT1 (Fig. 1A), miR-381 (Fig. 1B) and IGF1 (Fig. 1C–E) expression in ovarian granulosa cells of patients with PCOS was measured by RT-qPCR and Western blot analysis, and the results revealed that IGF1 and NEAT1 expression was increased and miR-381 expression was decreased in the PCOS group versus the non-PCOS group (all *P* < 0.05). To explore the mechanism of NEAT1/miR-381/IGF1 axis in PCOS, we applied Pearson test to analyze the relationship between NEAT1 and miR-381 expression, as well as that between miR-381 and IGF1 expression in PCOS, and the results showed (Fig. 1F, G) that in ovarian granulosa cells of patients with PCOS, NEAT1 expression was negatively correlated with miR-381 expression (r = − 0.68, *P* < 0.01), and miR-381 expression was negatively correlated with IGF1 expression (r = − 0.73, *P* < 0.01).

**Fig. 1:** NEAT1 and IGF1 expression are high and miR-381 expression is low in patients with PCOS. **A** NEAT1, expression in ovarian granulosa cells of patients with PCOS by RT-qPCR; **B** miR-381 expression in ovarian granulosa cells of patients with PCOS by RT-qPCR; **C** IGF1 mRNA expression in ovarian granulosa cells of patients with PCOS by RT-qPCR; **D** IGF1 protein bands in ovarian granulosa cells of patients with PCOS; **E** IGF1 protein expression in ovarian granulosa cells of patients with PCOS by Western blot analysis; **F** Pearson analyzed the relationship between NEAT1 and miR-381 in ovarian granulosa cells of patients with PCOS; **G** Pearson analyzed the relationship between miR-381 and IGF1 in ovarian granulosa cells of patients with PCOS; non-PCOS group = 108; PCOS group = 92. In **A**–**C**, the horizontal lines represent the average value, and whiskers represent the standard deviation. The data are all measurement data, expressed as mean ± standard deviation, and the *t* test was used for statistical analysis between the two groups. Pearson analysis was used for correlation analysis

### NEAT1 binds with miR-381 to target IGF1

To further analyze the relationship between NEAT1 and miR-381, and that between miR-381 and IGF1 in PCOS, binding sites between NEAT1 and miR-381 were analyzed and the pmirGLO-NEAT1-WT and pmirGLO-NEAT1-Mut plasmids were constructed (Fig. 2A). Dual luciferase reporter gene assay indicated that miR-381 mimic decreased the luciferase activity of the pmirGLO-NEAT1-WT vector while failed to reduce that of pmirGLO-NEAT1-Mut vector (Fig. 2B). RNA pull-down assay showed that the enrichment level of NEAT1 was increased in the Bio-miR-381-WT group by comparison with the Bio-NC group and Bio-miR-381-Mut group (both *P* < 0.05) (Fig. 2C). This result indicated that miR-381 was a target of NEAT1.

**Fig. 2:** NEAT1 binds with miR-381, and IGF1 is the direct target gene of miR-381 in PCOS rats. **A** The putative complementary binding sites of miR-381 and NEAT1; **B** Luciferase activity assay verified the targeting relationship between NEAT1 to miR-381; **C** RNA pull-down assay was used to detect the enrichment of NEAT1 by miR-381; **D** The putative complementary binding sites of miR-381 and IGF1; **E** Luciferase activity assay verified the targeting relationship between miR-381 and IGF1; **F** NEAT1 expression in ovarian tissues of PCOS rats by RT-qPCR; **G** miR-381 expression in ovarian tissues of PCOS rats by RT-qPCR; **H** IGF1 mRNA expression in ovarian tissues of PCOS rats by RT-qPCR; **I** IGF1 protein bands in ovarian tissues of PCOS rats by Western blot analysis; **J** IGF1 protein expression in ovarian tissues of PCOS rats by Western blot analysis; In **A**–**E**, N = 3. In **F**–**J**, n = 8. The data are all measurement data, expressed as mean ± standard deviation, the *t* test was used for statistical analysis between the two groups, and one-way ANOVA and Tukey’s post hoc test were used for statistical analysis among multiple groups. *P < 0.05 vs. the normal group; #*P* < 0.05 vs. the sh-NC group

The binding sites of miR-381/IGF1 were searched out (Fig. 2D) and miR-381 mimic reduced the luciferase activity of ovarian granulosa cells transfected with IGF1-WT, while caused no change in the ovarian granulosa cells transfected with IGF1-Mut (Fig. 2E), showing that IGF1 was the direct target gene of miR-381.

To explore the specific mechanism of NEAT1/miR-381/IGF1 axis involved in PCOS, we used DHEA to induce a PCOS rat model. NEAT1 (Fig. 2F), miR-381 (Fig. 2G), IGF1 (Fig. 2H–J) expressions in ovarian tissues of PCOS rats were detected. The results showed NEAT1 and IGF1 expression was enhanced while miR-381 expression was impaired in ovarian tissues of rats in the DHEA group versus the normal group (all *P* < 0.05). In contrast to the sh-NC group, NEAT1 and IGF1 expression was decreased and miR-381 expression was increased in the sh-NEAT1 group (all *P* < 0.05).

### Silenced NEAT1 promotes FSH and suppresses T, E2 and LH production in PCOS rats

FSH and LH are secreted by pituitary glands to promote the development and maturation of follicular cells. Hypothalamic gonadotropin releasing hormone and ovarian estrogen jointly regulate the process [23]. In this paper, the production of E2, P4, T, FSH and LH was determined by ELISA. It was presented that the production of FSH was reduced, while that of T, E2 and LH was increased (all *P* < 0.05), and P4 showed no altered change (*P* > 0.05) in the DHEA group in contrast to the normal group. In contrast to the sh-NC group, the production of FSH was increased while that of T, E2 and LH was decreased (all *P* < 0.05), and P4 production showed no change (*P* > 0.05) in the sh-NEAT1 group (Fig. 3A–E).

**Fig. 3:** Silenced NEAT1 promotes FSH and suppresses T, E2 and LH production in PCOS rats. **A** E2 production in serum in PCOS rats after down-regulation of NEAT1; **B** P4 production in serum in PCOS rats after down-regulation of NEAT1; **C** T production in serum in PCOS rats after down-regulation of NEAT1; **D** FSH production in serum in PCOS rats after down-regulation of NEAT1; **E** LH production in serum in PCOS rats after down-regulation of NEAT1. n = 8. The data are all measurement data, expressed as mean ± standard deviation, *P < 0.05 vs. the normal group; #*P* < 0.05 vs. the sh-NC group, and one-way ANOVA and Tukey’s post hoc test were used for statistical analysis. E2 for estradiol; P4 for progesterone; T for testosterone; FSH for follicle stimulating hormone; LH for luteinizing hormone

### Silenced NEAT1 alleviates pathological changes in PCOS rats

PCOS is pathologically manifested as abnormal follicular development and metabolic and endocrine disorders. To further observe histopathological changes in PCOS rats, HE staining was performed to observe that the ovarian granulosa cells in the normal group were intact and arranged regularly. Some fresh corpus luteum and follicles were observed, and no pathological phenomena such as cell necrosis, degeneration and inflammatory infiltration occurred. In the DHEA group and the sh-NC group, the ovary of the rats showed diffuse cystic severe dilatation and typical polycystic changes. Many small follicles dilated into large follicles, few corpus luteum and mature follicles and incomplete granulosa cells were observed. The ovary of rats in the sh-NEAT1 group showed diffuse cystic mild-moderate dilatation, with a small amount of corpus luteum and atresia follicles (Fig. 4A). Moreover, the number of mature follicles and corpus luteum in ovarian tissues of rats in the DHEA group was obviously lower than that in the normal group (*P* < 0.05). In contrast to the sh-NC group, the number of mature follicles and corpus luteum was increased in the sh-NEAT1 group (*P* < 0.05) (Fig. 4B, C).

**Fig. 4:** Silenced NEAT1 alleviates pathological changes in PCOS rats. **A** HE staining was used for observation of the pathological changes of ovary in PCOS rats after down-regulation of NEAT1 (Scale bar = 100 um); **B** The number of mature follicles in ovarian tissues of PCOS rats after down-regulation of NEAT1; **C** The number of corpus luteum in ovarian tissues of PCOS rats after down-regulation of NEAT1. n = 8. The data are all measurement data, expressed as mean ± standard deviation, *P < 0.05 vs. the normal group; #*P* < 0.05 vs. the sh-NC group, and one-way ANOVA and Tukey’s post hoc test were used for statistical analysis

### Silenced NEAT1 inhibits ovarian granulosa cell apoptosis in PCOS rats

Stimulated by FSH, the gap junction between granulosa cells and oocytes is in an open state and molecular substances enter the oocyte in large quantities before LH production reaches the peak. The apoptosis of granulosa cells directly affects the development of oocytes, which may be the result of granulosa cells transmitting apoptosis information to oocytes [24, 25]. TUNEL assay was used to detect the apoptosis of granulosa cells, and the outcome showed that in contrast to the normal group, the apoptotic index of ovarian granulosa cells in the DHEA group increased obviously (*P* < 0.05), and the apoptotic cells were deeply stained. In contrast to the sh-NC group, the apoptotic index of ovarian granulosa cells was decreased in the sh-NEAT1 group (*P* < 0.05), and the apoptotic cells were lightly stained (Fig. 5A, B).

**Fig. 5:** Silenced NEAT1 inhibits ovarian granulosa cell apoptosis in PCOS rats. **A** TUNEL assay was used to detect the apoptosis of ovarian granulosa cells in PCOS rats after down-regulation of NEAT1 (Scale bar = 50 μm); **B** Apoptotic index of ovarian granulosa cells in PCOS rats after down-regulation of NEAT1; **C** Protein bands of Cleaved caspase-3, caspase-3, Bax and Bcl-2 in PCOS rats after down-regulation of NEAT1. **D** Cleaved caspase-3/caspase-3 protein expression in PCOS rats after down-regulation of NEAT1 detected by Western blot analysis. **E** Bax/Bcl-2 protein expression in PCOS rats after down-regulation of NEAT1 detected by Western blot analysis; n = 8. The data are all measurement data, expressed as mean ± standard deviation, *P < 0.05 vs. the normal group; #*P* < 0.05 vs. the sh-NC group, and one-way ANOVA and Tukey’s post hoc test were used for statistical analysis

Western blot analysis showed that Cleaved caspase-3/caspase-3 ratio was increased while Bcl-2/Bax ratio was decreased in the DHEA group versus the normal group (all *P* < 0.05). The sh-NEAT1 group had reduced Cleaved caspase-3/caspase-3 ratio and elevated Bcl-2/Bax ratio versus the sh-NC group (all *P* < 0.05) (Fig. 5C–E).

### NEAT1 and IGF1 expression is elevated, and miR-381 expression is decreased in ovarian granulosa cells from PCOS rats

To further explore the specific mechanism of NEAT1/miR-381/IGF1 axis in PCOS at the cellular level, we extracted ovarian granulosa cells from PCOS rats. We performed HE staining and immunochemistry of FSHR to identify the extracted cells. HE staining showed that the ovarian granulosa cells were polygonal, the cytoplasm was reddish, and the nuclei were dark blue (Additional file 1: Fig. S1A).

FSHR was specifically expressed in ovarian granulosa cells and its expression was detected by immunochemistry. It was tested that FSHR positive staining (brown) was localized in the cytoplasm of the cells, and the nucleus was dark blue. The positive rate of FSHR exceeded 90%, therefore, the extracted ovarian granulosa cells could be applied to the cell experiments (Additional file 1: Fig. S1B). Then, we intervened NEAT1 and miR-381 expression in the ovarian granulosa cells from PCOS rats. NEAT1 expression levels in ovarian granulosa cells were assessed by RT-qPCR and Western blot analysis (Fig. 6A). The results showed that in contrast to the sh-NC group, NEAT1 expression was decreased in the sh-NEAT1 group (*P* < 0.05). Versus the pc-NC group, NEAT1 expression was increased in the pc-NEAT1 group (*P* < 0.05), suggesting successful intervention in NEAT1 expression in ovarian granulosa cells from PCOS rats.

**Fig. 6:** NEAT1 and IGF1 expression is elevated, and miR-381 expression is repressed in ovarian granulosa cells from PCOS rats. **A** NEAT1 expression in ovarian granulosa cells from PCOS rats after transfection by RT-qPCR; **B** miR-381 expression in ovarian granulosa cells from PCOS rats after transfection by RT-qPCR; **C** IGF1 mRNA expression in ovarian granulosa cells from PCOS rats after transfection by RT-qPCR; **D** IGF1 protein bands in ovarian granulosa cells from PCOS rats after transfection by Western blot analysis; **E** IGF1 protein expression in ovarian granulosa cells from PCOS rats after transfection by Western blot analysis N = 3. The data are all measurement data, expressed as mean ± standard deviation, *P < 0.05 vs. the sh-NC group; ^*P* < 0.05 vs. the pc-NC group; #*P* < 0.05 vs. the mimic NC group, &*P* < 0.05 vs. the pc-NEAT1 + mimic NC group, and one-way ANOVA and Tukey’s post hoc test were used for statistical analysis

Then, we detected the expression levels of miR-381 (Fig. 6B) and IGF1 (Fig. 6C–E) in the ovarian granulosa cells from PCOS rats by RT-qPCR and Western blot analysis. The results showed that in contrast to the sh-NC group, IGF1 expression was decreased, and miR-381 expression was increased in the sh-NEAT1 group (all *P* < 0.05). In contrast to the mimic NC group, IGF1 expression was decreased and miR-381 expression was increased in the miR-381 mimic group (both *P* < 0.05). Compared with the pc-NEAT1 + mimic NC group, IGF1 expression was decreased and miR-381 expression was increased in the pc-NEAT1 + miR-381 mimic group (both *P* < 0.05).

### Silenced NEAT1 or elevated miR-381 promotes proliferation of ovarian granulosa cells from PCOS rats

Ovarian granulosa cell proliferation plays a vital role in PCOS. Ovarian granulosa cell proliferation after transfection was detected via CCK-8, colony formation assays and RT-qPCR. The results showed that in contrast to the sh-NC group, mimic NC group and pc-NEAT1 + mimic NC group, respectively, the cell proliferation at 48–72 h, the number of colonies, as well as proliferating cell nuclear antigen (PCNA) and Cyclin D1 mRNA expression were increased in the sh-NEAT1 group, miR-381 mimic group and pc-NEAT1 + miR-381 mimic group (all *P* < 0.05) (Fig. 7A–D).

**Fig. 7:** Cell proliferation is promoted by silenced NEAT1 or elevated miR-381 in ovarian granulosa cells from PCOS rats. **A** Difference in cell viability after transfection of ovarian granulosa cells from PCOS rats by CCK-8 assay; **B** PCNA and cyclin D1 mRNA expression in ovarian granulosa cells from PCOS rats by RT-qPCR; **C**, **D** Colony formation ability of ovarian granulosa cells from PCOS rats detected by colony formation assay; N = 3. The data are all measurement data, expressed as mean ± standard deviation, *P < 0.05 vs. the sh-NC group; #*P* < 0.05 vs. the mimic NC group, &*P* < 0.05 vs. the pc-NEAT1 + mimic NC group, and one-way ANOVA and Tukey’s post hoc test were used for statistical analysis

### Silenced NEAT1 or elevated miR-381 inhibits apoptosis of ovarian granulosa cells from PCOS rats

Ovarian granulosa cell apoptosis is essential in the progression of PCOS. Annexin V/PI assay showed that in contrast to the sh-NC, mimic NC and pc-NEAT1 + mimic NC groups, respectively, the apoptosis rate of cells was decreased in the sh-NEAT1, miR-381 mimic, and pc-NEAT1 + miR-381 mimic groups (all *P* < 0.05) (Fig. 8A, B).

**Fig. 8:** Cell apoptosis is inhibited by silenced NEAT1 or elevated miR-381 in ovarian granulosa cells from PCOS rats. **A** Apoptosis of ovarian granulosa cells from PCOS rats after transfection by flow cytometry; **B** Comparison of apoptosis rate of ovarian granulosa cells from PCOS rats after transfection; **C** Caspase-3 mRNA expression in ovarian granulosa cells from PCOS rats after transfection; **D** Bax mRNA expression in ovarian granulosa cells after transfection; **E** Bcl-2 mRNA expression in ovarian granulosa cells from PCOS rats after transfection; N = 3. The data are all measurement data, expressed as mean ± standard deviation, *P < 0.05 vs. the sh-NC group; #*P* < 0.05 vs. the mimic NC group, &*P* < 0.05 vs. the pc-NEAT1 + mimic NC group, and one-way ANOVA and Tukey’s post hoc test were used for statistical analysis

RT-qPCR demonstrated that in contrast to the sh-NC, mimic NC and pc-NEAT1 + mimic NC groups, Caspase-3 and Bax mRNA expression levels were decreased, and Bcl-2 mRNA expression level was elevated in the sh-NEAT1, miR-381 mimic and pc-NEAT1 + miR-381 mimic groups (all *P* < 0.05) (Fig. 8C–E).

### Overexpression of IGF1 impairs the biological activity of ovarian granulosa cells from PCOS rats induced by up-regulated miR-381

To further explore the effect of IGF1 on the function of ovarian granulosa cells from PCOS rats, rescue experiments were implemented to find that versus the mimic NC + pc-CON group, cell proliferation was enhanced, apoptosis was inhibited, PCNA, cyclin D1 and Bcl-2 mRNA expression was increased, caspase-3 and Bax mRNA expression was decreased in the miR-381 mimic + pc-CON group (all *P* < 0.05); compared with the miR-381 mimic + pc-CON group, cell proliferation was decreased, apoptosis was increased, PCNA, cyclin D1 and Bcl-2 mRNA expression was decreased, caspase-3 and Bax mRNA expression was increased in the miR-381 mimic + pc-IGF1 group (all *P* < 0.05) (Fig. 9A–H).

**Fig. 9:** Overexpression of IGF1 impairs the biological activity of ovarian granulosa cells from PCOS rats induced by up-regulated miR-381. **A** Overexpression of IGF1 in ovarian granulosa cells from PCOS rats; **B** Difference in cell viability after transfection of ovarian granulosa cells from PCOS rats by CCK-8 assay; **C**, **D** Colony formation ability of ovarian granulosa cells from PCOS rats detected by colony formation assay; **E** PCNA and cyclin D1 mRNA expression in ovarian granulosa cells from PCOS rats by RT-qPCR; **F**, **G** Apoptosis of ovarian granulosa cells from PCOS rats after transfection by flow cytometry; **H** Caspase-3, Bax and Bcl-2 mRNA expression in ovarian granulosa cells from PCOS rats after transfection by RT-qPCR; N = 3. The data are all measurement data, expressed as mean ± standard deviation, *P < 0.05 vs. the pc-CON + mimic NC group; #*P* < 0.05 vs. the miR-381 mimic + pc-CON group, and one-way ANOVA and Tukey’s post hoc test was used for statistical analysis

## Discussion

PCOS is a heterogeneous endocrine aberration in reproductive age women with high prevalence and socioeconomic costs [26, 27]. Extended estrogen excess or scarce of progesterone leads to atypical endometrial hyperplasia, PCOS women with endometrial hyperplasia bear higher risk of developing endometrial carcinoma than non-PCOS women [28]. Additionally, women with PCOS are also reported to own a high risk of obstetric complications including preeclampsia, gestational diabetes and preterm birth [29]. In the present study, we highlighted the role of NEAT1 in PCOS and its underlying mechanisms and found that downregulation of NEAT1 or upregulation of miR-381 stimulated ovarian granulosa cell proliferation and repressed apoptosis in PCOS rats through inhibiting IGF1.

The initial finding from our research showed that NEAT1 and IGF1 were highly expressed while miR-381 was lowly expressed in PCOS. In line with the results in our study, a recent study highlighted that NEAT1 expression tended to upregulate in PCOS [9]. Similarly, NEAT1 was upregulated in tissues and cells of PCOS [9]. Similar to our study, a prior study has revealed that miR-381 was decreased in EOC and restoring miR-381 impeded cancer progression [30]. Nevertheless, the expression of miR-381 in PCOS is seldom investigated. Also, the serum levels of IGF-1 have been found to be significantly elevated in women with PCOS relative to controls [15]. Except that, this present study also suggested that NEAT1 could function as a ceRNA to adsorb miR-381, and IGF1 was the direct target gene of miR-381. In fact, NEAT1 has been evidenced to mediate miR-381 [31] while the targeting relation between miR-381 and IGF1 requires further verification.

Next, we found that silenced NEAT1 promoted the production of FSH and suppressed that of T, E2 and LH in PCOS rats and inhibited apoptosis of ovarian granulosa cells. The family of apoptotic proteins (including Bcl-2, Bax and Cleaved caspase-3) is an important component of the apoptotic pathway [32, 33]. We have also found that silenced NEAT1 or elevated miR-381 promoted cell proliferation, PCNA and cyclin D1 expression. In line with our findings, it has been revealed that ectopic expression of NEAT1 stimulated the development of PCOS, and NEAT1 can enhance the proliferation of ovarian granulosa cells and arrest cell apoptosis [7, 9]. Meanwhile, a previous article also suggested that NEAT1 knockdown elevated cell sensitivity to paclitaxel (PTX) through inducing PTX-mediated apoptosis in vitro and in vivo [34]. On the other hand, miR-381 has been demonstrated to restrict colorectal cancer cell migration and invasion [35]. In vitro and in vivo assays in another study have demonstrated that miR-381 blocked the proliferative behavior of gastric cancer cells [36]. Besides, overexpressed miR-381-3p contributed to markedly improved spinal cord injury [37]. All these evidences conformed the positive role of depleted NEAT1 and restored miR-381 in the disease progression. As to the role of IGF1 in PCOS, a previous research has proved that it was up-regulated in PCOS and suppression of IGF1 partially alleviated PCOS, as reflected by reduced T and LH and increased FSH production, as well as enhanced proliferation and impaired apoptosis of granulosa cells [13]. Also, highly expressed IGF1 in PCOS could inhibit granulosa cell proliferation and promote cell apoptosis [38]. From another perspective, IGF1 downregulation could repress granulosa-like tumor cell proliferation and induce cell apoptosis in PCOS [39]. Anyway, the promoting role of suppressed IGF1 in PCOS is consistent with our research.

## Conclusion

In conclusion, our study has revealed that downregulation of NEAT1 or upregulation of miR-381 contributed to the promotion of granulosa cell proliferation and the repression of apoptosis in PCOS by inhibiting IGF1 expression. These results suggest that NEAT1/miR-381/IGF1 axis plays an essential part in the pathogenesis of PCOS. This research provides new possible molecular targets for the future treatments of PCOS, as well as a new theoretical basis for subsequent drug development. However, this study is partly limited to insufficiency of clinical investigations, which shall be further studied in the future.

## Supplementary Information

**Additional file 1: Fig. S1**. Identification of ovarian granulosa cells. A. HE staining of ovarian granulosa cells (scale bar: 25 μm); B. Identification of ovarian granulosa cells (FSHR, cellular immunochemistry; scale bar: 25 μm).

## Data Availability

Not applicable.
